# Antifungal Activity of* Lactobacillus* sp. Bacteria in the Presence of Xylitol and Galactosyl-Xylitol

**DOI:** 10.1155/2016/5897486

**Published:** 2016-05-12

**Authors:** Lidia Lipińska, Robert Klewicki, Elżbieta Klewicka, Krzysztof Kołodziejczyk, Michał Sójka, Adriana Nowak

**Affiliations:** ^1^Institute of Fermentation Technology and Microbiology, Faculty of Biotechnology and Food Sciences, Lodz University of Technology, Wolczanska 171/173, 90-924 Lodz, Poland; ^2^Institute of Chemical Technology of Food, Faculty of Biotechnology and Food Sciences, Lodz University of Technology, Stefanowskiego 4/10, 90-924 Lodz, Poland

## Abstract

Lactic acid fermentation is a natural method of antimicrobial food protection. Antagonistic activity of* Lactobacillus* sp. bacteria, taking part in this process, is directed mainly against the same or other microorganisms. In this work we determine the impact of the presence of xylitol and galactosyl-xylitol on the antagonistic activity of 60* Lactobacillus* sp. strains against indicator molds (*Alternaria alternata*,* Alternaria brassicicola*,* Aspergillus niger*,* Fusarium latenicum*,* Geotrichum candidum*, and* Mucor hiemalis*) and yeasts (*Candida vini*). We used double-layer method to select antifungal strains of* Lactobacillus* bacteria and poisoned medium method to confirm their fungistatic properties. Additionally, we examined the inhibition of* Alternaria brassicicola* by* Lactobacillus paracasei* ŁOCK 0921 cultivated with xylitol or galactosyl-xylitol directly on wild cherries. The presence of xylitol and its galactosyl derivative led to increase of spectrum of antifungal activity in most of the studied plant-associated lactobacilli strains. However, no single strain exhibited activity against all the indicator microorganisms. The antifungal activity of* Lactobacillus* bacteria against molds varied considerably and depended on both the indicator strain and the composition of the medium. The presence of xylitol and galactosyl-xylitol in the growth medium is correlated with the antifungal activity of the studied* Lactobacillus* sp. bacteria against selected indicator molds.

## 1. Introduction

Lactic acid fermentation constitutes one of the oldest methods of protecting food from undesirable microflora. However, lactic acid bacteria (LAB) generate antimicrobial compounds inhibiting the growth of related species and show low antagonistic activity towards fungi, the most widespread food spoilage factors. To improve the antifungal effect of* Lactobacillus* sp., genus belonging to LAB, researchers modify their growth medium to stimulate metabolism towards production of antifungal compounds [1–3].

Our preliminary studies confirmed that polyols (glycerol, lactitol, erythritol, sorbitol, and mannitol) may enhance the antifungal activity of LAB [2]. Furthermore, some polyols such as sorbitol, xylitol, erythritol, and lactitol are applied in the food industry and benefit human health [4]. An example of such compound is xylitol, a five-carbon polyol [5], which has a GRAS status (Generally Recognized as Safe) and is applied in pharmaceutical and food industry as an antidiabetic substitute for sucrose [6]. As a low-calorie compound, xylitol is added to sweets [7–9], chewing gum, toothpaste, and dental sealants due to its anticaries properties [10–13]. However, the effect of xylitol and its galactosyl derivative on antifungal properties of LAB has not been studied in detail. Besides, galactosyl-xylitol represents a modern prebiotic and can improve condition of gastrointestinal track.

The objective of our study was to determine the antagonistic activity of 60* Lactobacillus *sp. strains in the presence of xylitol and its galactosyl derivative (galactosyl-xylitol) against selected food-contaminating fungi.

## 2. Materials and Methods

### 2.1. Bacteria of the Genus* Lactobacillus *and Indicator Fungal Strains

The study material consisted of 60 bacterial (*Lactobacillus *sp.) and 8 fungal strains deposited with the Pure Cultures Collection of Industrial Microorganisms of the Institute of Fermentation Technology and Microbiology, Lodz University of Technology (ŁOCK 105).

Examined* Lactobacillus *sp. strains were divided into four groups depending on the species (*L. acidophilus *strains and* L. casei/paracasei *strains) and origin (plant strains and strains isolated from humans). First group consisted of 20 strains of* L. acidophilus* designated as 7, 0840, 0842, 0926–0939, and 0941–0943; second one consisted of 23 strains of* L. casei/paracasei*:* L. casei* 0848, 0901–0907, 0909–0911, and 0919, Paris, NCDO206, and* L. paracasei* 0912, 0913, 0917, 0918, 0920–0922, 0924, and 0985; third group consisted of 13 plant-associated strains:* L. plantarum *0981, 0982, 0989, and 0990,* L. pentosus *0979 and 0991,* L. brevis *0944, 0980, 0983, and 0984,* L. helveticus*,* L. delbrueckii *0854, and* L. casei *1020; and the last one consisted of 4 strains isolated from humans:* L. casei *0919,* L. delbrueckii *0987,* L. mucosae* 0988, and* L. rhamnosus *0908.

*Bacteria*.* L. acidophilus*,* L. casei*,* L. helveticus*,* L. paracasei*, and* L. rhamnosus* were incubated at 37°C under aerobic conditions, the strains isolated from humans at 37°C in the presence of CO_2_, and the plant-associated strains at 30°C under aerobic conditions. All bacteria were stored at −20°C in 20% (v/v) glycerol. 

*The Yeasts Candida vini 0008 and 0009 and the Molds*.* Mucor hiemalis* 0519,* Geotrichum candidum* 0511,* Alternaria alternata* 0409,* Alternaria brassicicola* 0412,* Aspergillus niger* 0433, and* Fusarium latenicum* 0508 constituted the indicator microorganisms. They were kept at 4°C on Sabouraud 4%-dextrose agar slants (Merck).

### 2.2. Synthesis of the Galactosyl Derivative of Xylitol

The galactosyl derivative of xylitol was obtained by enzymatic transglycosylation using *β*-galactosidase EC 3.2.1.23 from* Kluyveromyces lactis* (Novozymes A/S, Bagsvaerd, Denmark). The procedure for the synthesis of galactosyl-xylitol was described by Klewicki [14].

### 2.3. Selection of Antifungal* Lactobacillus *Strains in the Presence of Xylitol and Galactosyl-Xylitol

The antagonistic activity of* Lactobacillus *bacteria against indicator fungi was tested by the double-layer method. 24-hour cultures of a given* Lactobacillus* sp. strain were drop plated (with droplets of 10 *μ*L) on MRS agar medium (Merck or BTL) with or without 10 g of xylitol, galactosyl-xylitol, or galactose per liter. The control group consisted of MRS agar plates (Merck) without LAB cultures. After 18–24 hours the plates were overlaid with Sabouraud 4%-dextrose agar (Merck) inoculated with an indicator fungal strain (10^5^–10^6^ spores mL^−1^). We measured inhibition zones of the indicator strain around colonies of* Lactobacillus *sp. after 24–72 hours (30°C, aerobic conditions). The results were given as fungal inhibition diameters minus the diameter of* Lactobacillus* sp. colonies.

### 2.4. Antifungal Activity Assay on Wild Cherries (*Prunus avium*)

Antifungal effect of sterile supernatants after 30 hours of lactic acid fermentation of* Lactobacillus paracasei *ŁOCK 0921 in the presence of xylitol or galactosyl-xylitol against* Alternaria brassicicola *was estimated. Examined bacterial strain was chosen based on the results of screening of antifungal lactobacilli. Indicator microorganisms of the genus* Alternaria *were chosen because they are frequently isolated from wild cherries [15] and they can produce mycotoxins [16]. Wild cherries (average weight 4.8–5.3 g) were washed and soaked in sterile distilled water and left to dry for 30 minutes under sterile conditions (laminar flow chamber BioHazard type II). The fruits (wild cherries) were treated with* A. brassicicola* (suspension of conidia in 0.85% NaCl, 1*∗*10^5^ cells·mL^−1^) by dissecting needle (0.5 mm in diameter, one puncture per fruit). Then, cell-free supernatant (10 *μ*L, 20 *μ*L, and 100 *μ*L) of* L. paracasei *ŁOCK 0921, cultivated with 1% (w/v) xylitol or galactosyl-xylitol (48 hours, 37°C), was dropped in infected fruit. Corresponding experiments were conducted with cell-free supernatant of* L. paracasei *ŁOCK 0921 in the growing medium with glucose only, followed by the medium with galactose alone. The mold-inoculated wild cherries were incubated for 10 days at 23.4 ± 0.2°C. Incubation time has been prolonged on the grounds of using temperature lower than in other studies, typical for storing wild cherries, and to check the appearance of the possible secondary growth of indicator molds.

### 2.5. Antifungal Effect of Postcultivation Supernatant of* Lactobacillus *sp. Poisoned Media Method

We modified poisoned media method described by Manici et al. [17]. Mold* Alternaria brassicicola* was cultivated on Petri plates with Sabouraud 4%-dextrose agar (Merck) supplemented with 10, 20, 30, 50, and 70% (v/v) cell-free supernatant obtained after 30 hours of lactic acid fermentation of* Lactobacillus pentosus *ŁOCK 0979, strain with antifungal activity towards most indicator fungi, or* Lactobacillus paracasei *ŁOCK 0921, used in the study on wild cherries and shown in Figure 2, with 1% (w/v) xylitol or galactosyl-xylitol. Molds were incubated for 8 days (30°C, aerobic conditions). We measured the diameter of their colonies every day and estimated linear growth index using the following formula:

(1) $$\begin{array}{c} T=\frac{A}{D}+\frac{b_{1}}{d_{1}}+\cdots +\frac{b_{x}}{d_{x}}, \end{array}$$

where *T* is linear growth index; *A* is diameter of fungal colony [mm]; *D* is time [days]; *b*_1_,…, *b*_*x*_ are increase of fungal colony [mm]; *d*_1_,…, *d*_*x*_ are time between measurements.

The fungistatic activity of cell-free supernatant was estimated according to Abbot's formula [18, 19]:

(2) $$\begin{array}{c} I=\frac{\left(K-A\right)}{K}*100\%, \end{array}$$

where *I* is inhibition/stimulation rate according to Abbot's formula; *K* is diameter of fungal colony on control plate; *A* is diameter of fungal colony on experimental plate.

### 2.6. Statistical Analysis

The tests were done in triplicate. The experimental data is expressed as mean ± standard deviation (SD). One-way analysis of variance (ANOVA) and the Bonferroni* post hoc* test (*p* ≤ 0.05) were applied to find differences between groups.

## 3. Results and Discussion

### 3.1. Screening of Antifungal* Lactobacillus *sp. Strains

Antifungal activity of examined bacterial strains depends on growth medium and fungal indicator strain. None of the tested* Lactobacillus *sp. strains appreciably inhibited growth of yeasts* Candida vini*. We observed slight inhibition (1.0 ± 0.0 mm) of indicator yeasts by three strains of lactobacilli:* L. mucosae *0988,* L. delbrueckii *0987, both isolated from human, and plant-associated* L. pentosus *0979.

*Lactobacillus *sp. bacteria poorly suppressed three out of six testing mold strains. Growth of the most resistant mold,* Geotrichum candidum* 0511, was inhibited only in the presence of xylitol in the range from 1.3 to 3.1 mm (Figure 1(c)). Origin of lactobacilli strains had no significant impact on their antagonistic activity against* G. candidum*. Growth inhibition of* A. niger *(Figure 1(a)) and* M. hiemalis *(Figure 1(e)) was moderate. Plant-associated bacterial strains showed the strongest antagonistic effect against* Aspergillus niger *(0.9–6.3 mm of the inhibition zone diameter). Growth of this mold was not suppressed in the sample containing galactose in MRS agar (BTL, without glucose). Mold* M. hiemalis* was the most inhibited in the control sample and in the presence of xylitol (especially by the plant-associated strains) and galactosyl-xylitol (by both plant-associated and human strains) and the least inhibited in the presence of galactose (Figure 1(e)). Molds* A. alternata *(Figure 1(b)),* A. brassicicola *(Figure 1(d)), and* F. latenicum* (Figure 1(f)) exhibited high sensitivity to* Lactobacillus* sp. bacteria in the control samples. However, the presence of xylitol and galactosyl-xylitol increased their susceptibility to products of lactic acid fermentation. The growth of* A. brassicicola *was completely inhibited in the presence of galactosyl-xylitol.

Among the studied fungal indicators, the* A. alternata* was the most susceptible to LAB metabolites. In turn, in the presence of galactose that strain was only slightly inhibited, mostly by the plant-associated* Lactobacillus *strains. In the case of the antagonism of* L. acidophilus* and* L. casei/paracasei *against the mold* A*.* brassicicola*, the inhibition zones increased in the presence of galactose, but not as much as in the presence of galactosyl-xylitol (Figure 1(d)). In this study,* Lactobacillus *bacteria isolated from plant and human sources have shown the strongest average antifungal activity against indicator molds except* G. candidum.* Crowley et al. [20] described similar correlations between lactobacilli origin and their antifungal effect. They screened 70 samples isolated from various sources, isolated LAB, and observed the strongest antifungal effect of* Lactobacillus* sp. obtained from plants and humans. Strong correlation between origin of lactobacilli and their antagonistic activity against fungi was not found in other studies. In our review article [21] current knowledge about antifungal activity of lactobacilli is presented. Many* Lactobacillus *species have antifungal activity against proper mold or even yeast; however this activity is usually poor or moderate. Lactobacilli species, which are best described as producers of antifungal compounds, are* L. acidophilus*,* L. brevis*,* L. casei*,* L. fermentum*,* L. plantarum*,* L. reuteri*,* L. rhamnosus*, and* L. sakei*.

The primary goal of our study was to collate the antifungal activity of lactobacilli in different medium. We observed strong correlation between the presence of xylitol and galactosyl-xylitol and the antagonistic activity of LAB isolated from different sources. Figure 2 presents the significantly disparate results of inhibition zones of* A. brassicicola* around* Lactobacillus* sp. colonies cultivated in the medium containing xylitol or galactosyl-xylitol and various carbon sources: glucose or galactose.

Table 1 shows the antagonistic activity of selected* Lactobacillus* sp. strains against the indicator fungi on all the tested media, MRS agar with glucose, galactose, both glucose and galactose, xylitol, or galactosyl-xylitol. We selected* Lactobacillus* strains with high inhibitory activity against a given indicator fungal strain. The bacterial strain with the widest spectrum of antifungal activity was* L. acidophilus *0927, strongly affecting* A. alternata *in the presence of xylitol and galactosyl-xylitol and inhibiting* A. brassicicola *in all of the tests but affecting* G. candidum *only in the presence of xylitol (inhibition zone of 11.0 mm). The molds* F. latenicum *and* M. hiemalis *were most inhibited by* L. brevis* 0980, while mold* A. niger *was inhibited by* L. plantarum *0982.

### 3.2. Antifungal Activity Assay of* Lactobacillus *sp. Supernatants on Wild Cherries

We observed inhibition of* Alternaria brassicicola *on wild cherries treated with cell-free supernatant after fermentation of* Lactobacillus paracasei *ŁOCK 0921 in the presence of xylitol. The presence of galactosyl-xylitol also affected antifungal activity of tested bacterial strain but volume of 10 *μ*L of cell-free supernatant was insufficient to inhibit the growth of* A. brassicicola.* However, examined mold was totally inhibited with 20 and 100 *μ*L, while the volume of 10 *μ*L was too low (Figure 3). After the fermentation of* Lactobacillus paracasei* ŁOCK 0921 in the presence of glucose (Figure 3(c)) or galactose (Figure 3(d)) the cell-free supernatant has not shown antifungal activity against* A. brassicicola* at any volume; Figures 3(c) and 3(d) present the highest volume (100 *μ*L) of cell-free supernatant.

### 3.3. Fungistatic Effect of Cell-Free Supernatant after Lactic Acid Fermentation with Xylitol or Galactosyl-Xylitol

We cultivated* Alternaria brassicicola* on Petri dishes with 10, 20, 30, 50, or 70% (v/v) of cell-free supernatant after lactic acid fermentation of* Lactobacillus pentosus *0979 and* Lactobacillus paracasei *0921 in the presence of xylitol or galactosyl-xylitol. We have measured mold colony diameters for 8 days and estimated linear growth index (*T*) and inhibition/stimulation rate (*I*) according to Abbot's formula (Table 2).

In the presence of xylitol and galactosyl-xylitol the cell-free supernatant of* L. pentosus *0979 which was placed in fungal medium has shown absolute inhibition of* A. brassicicola* in all tested cases.* L. paracasei *0921, mentioned in study on wild cherries and in Figure 2, demonstrated similar effect in the presence of galactosyl-xylitol, but only moderate fungistatic effect cultivated in the presence of xylitol (10% and 20% of supplementation).

The antifungal activity of* Lactobacillus *bacteria depends on the growth medium and is distinctive for all studied fungal species [22]. Klewicka and Klewicki [3] investigated the growth and metabolism of lactic acid bacteria in the presence of some polyols and their galactosyl derivatives. They found that LAB grew poorly in the presence of xylitol; meanwhile in the presence of galactosyl-xylitol their growth was comparable to the controls. This implies that the studied LAB efficiently use galactosyl-polyols to hydrolyze galactosyl bonds enzymatically and to cleave the galactose molecule. In the case of galactosyl-polyol fermentation, galactose is the first saccharide metabolized by the tested bacteria. The amounts of lactic and acetic acids synthesized by lactobacilli in the presence of galactosyl-xylitol were similar to or lower than those observed in the glucose-containing control samples [3]. It may therefore be inferred that the antagonistic effect of* Lactobacillus* sp. bacteria in the presence of xylitol and galactosyl-xylitol results from xylitol metabolism. It may also be assumed that in the presence of polyols bacterial metabolism is directed towards effective synthesis of some secondary metabolites with antifungal properties.

Antifungal activity is linked to the synthesis of specific metabolites including low molecular weight peptides, such as reuterin isolated from* Lactobacillus reuteri* (MW 148 Da) [23], 3-hydroxy fatty acids [24], phenyllactic acid [25], and cyclic dipeptides [26]. Our preliminary studies suggest that antifungal effect of tested lactobacilli is probably correlated with acids production, especially phenyllactic acid, or with synergistic effect of acids and other antifungal compounds [data not shown]. Almståhl et al. [27] examined the metabolism of polyols, including xylitol, by selected bacterial strains. They isolated* Lactobacillus *sp. strains,* L. fermentum*,* L. casei*,* L. rhamnosus*,* L. salivarius*,* L. acidophilus*, and* L. gasseri*, as well as some unidentified strains, from the human oral cavity. Subsequently, they studied the ability of bacterial strains to ferment sugars (glucose, fructose, and sucrose) and polyols (mannitol, sorbitol, and xylitol). It was found that the bacterial strains grew more vigorously in media containing saccharides than in those containing polyols; also following lactic acid fermentation pH was lower in the former than in the latter [27]. Sugar fermentation led to lower pH as if during that process bacteria generated more lactic acid and other organic acids than during polyol fermentation. A similar correlation between the presence of polyols in the growth media and the metabolism of LAB was observed by Magnusson [26], who reported increased antifungal activity of* Lactobacillus coryniformis *in the presence of glycerol in the growth medium.

In our hypothesis, the use of xylitol or galactosyl-xylitol, instead of chemical preservatives, can be an alternative method to inhibit the growth of fungi in fermented food. Elucidation of the mechanism antagonistic activity of* Lactobacillus *sp. in the presence of xylitol and its galactosyl derivative is a promising avenue of research. Therefore, in the further studies we will focus our attention on the identification of specific lactic acid fermentation products with antifungal properties generated in the presence of polyols and their galactosyl derivatives.

## 4. Conclusions 

Antagonistic activity of investigated* Lactobacillus *sp. strains depends on both growth media and indicator strains of fungi. None of the bacterial strains demonstrated a wide spectrum of antagonistic activity against the indicator microorganisms, but some of them inhibited the growth of individual fungal strains in the presence of appropriate substrates. Moreover, molds are more susceptible to the presence of lactic acid bacteria and xylitol or galactosyl-xylitol than yeasts. Most of tested lactic acid bacteria have an antifungal effect only in the presence or xylitol or galactosyl-xylitol and have shown lower or no antifungal effect in the presence of glucose and galactose only. Antifungal activity assays of LAB supernatants on wild cherries and using poisoned media method confirmed that xylitol and galactosyl-xylitol can enhance antifungal properties of tested lactobacilli.

## Figures and Tables

**Figure 1:** Inhibition zones of indicator fungal strains caused by* Lactobacillus* sp. in the presence of xylitol, galactosyl-xylitol, and galactose.

**Figure 2:** Antagonistic activity of selected* Lactobacillus* bacteria strains against* A. brassicicola* in (a) the control sample without xylitol; (b) the control sample with only xylitol; (c)* Lactobacillus *sp. without xylitol; (d)* Lactobacillus *sp. with xylitol; (e)* Lactobacillus *sp. and galactosyl-xylitol; (f)* Lactobacillus *sp. and galactose with glucose; (g)* Lactobacillus *sp. and galactose without glucose. LAB strains: “172”* L. acidophilus *0926, “62”* L. paracasei *0921, “–”* L. paracasei *0917, and “291”* L. casei *0904.

**Figure 3:** Inhibition of* Alternata brassicicola *on wild cherries after 10 days of incubation with 10, 20, or 100 *μ*L cell-free supernatant after lactic acid fermentation by* Lactobacillus paracasei *ŁOCK 0921 in the presence of glucose (c), galactose (d), glucose + xylitol (e), or glucose + galactosyl-xylitol (f); (a) negative control (without molds); (b) positive control (infected by molds).

**Table 1:** Inhibition zones of indicator fungal strains caused by selected *Lactobacillus* sp. strains which have the strongest antagonistic activity against proper mold.

Strains of LAB	LAB medium	Diameter of inhibition zone of indicator molds caused by selected LAB [mm] ± SD^1^					
		*A. niger*	*A. alternata*	*A. brassicicola*	*F. latenicum*	*G. candidum*	*M. hiemalis*
*L. acidophilus *0927	Control	0.5 ± 0.7^a^	ND	19.0 ± 1.4^a^	16.0 ± 1.4^a^	—	3.5 ± 0.7^a^
	Xylitol	0.5 ± 0.7^a^	>90^a^	5.0 ± 1.4^b^	12.5 ± 0.7^b^	11.0 ± 0.0	6.0 ± 0.0^b^
	Galactosyl-xylitol	2.0 ± 0.0^b^	>90^a^	>90^c^	>90^c^	—	3.0 ± 0.0^a^
	Galactose + glucose	—	14.0 ± 0.0^b^	>90^c^	30.0 ± 0.7^d^	—	—
	Galactose	—	14.0 ± 0.0^b^	>90^c^	14.0 ± 0.0^ab^	—	—

*L. acidophilus* 0932	Control	—	—	8.0 ± 2.5^a^	18.0 ± 2.8^a^	—	—
	Xylitol	—	24.0 ± 0.0^a^	—	2.0 ± 0.0^b^	—	—
	Galactosyl-xylitol	—	>90^b^	>90^b^	>90^b^	—	3.0 ± 0.0
	Galactose + glucose	—	—	—	3.0 ± 0.0^b^	—	—
	Galactose	—	—	—	—	—	—

*L. acidophilus* 0937	Control	—	10.0 ± 0.0^a^	19.0 ± 4.2^a^	1.0 ± 0.0^a^	—	—
	Xylitol	8.0 ± 2.8	30.0 ± 0.0^b^	ND^b^	11.0 ± 1.4^b^	—	2.0 ± 0.0
	Galactosyl-xylitol	—	—	>90^c^	—	—	—
	Galactose + glucose	—	2.0 ± 0.0^c^	—	0.5 ± 0.0^a^	—	—
	Galactose	—	—	—	—	—	—

*L. brevis *0944	Control	—	25.0 ± 4.2^a^	1.5 ± 0.7^a^	5.0 ± 1.4^a^	—	4.0 ± 1.4^a^
	Xylitol	8.0 ± 0.0^a^	24.0 ± 0.0^a^	ND	18.0 ± 0.0^b^	15.5 ± 0.0^a^	7.5 ± 2.1^a^
	Galactosyl-xylitol	4.0 ± 0.0^b^	>90^b^	>90^b^	>90^c^	—	6.0 ± 0.0^a^
	Galactose + glucose	—	13.0 ± 0.0^c^	>90^b^	>90^c^	—	2.0 ± 0.0^b^
	Galactose	—	11.0 ± 0.0^d^	4.0 ± 0.0^c^	11.0 ± 0.0^d^	—	2.0 ± 0.0^b^

*L. brevis *0980	Control	—	ND	4.5 ± 0.7^a^	10.5 ± 0.7^a^	8.0 ± 0.0	8.0 ± 0.0^a^
	Xylitol	18.5 ± 2.1^a^	>90^a^	6.5 ± 0.7^a^	15.5 ± 0.7^b^	—	15.0 ± 7.2^ab^
	Galactosyl-xylitol	3.0 ± 0.0^b^	>90^a^	>90^b^	>90^c^	—	9.0 ± 0.0^b^
	Galactose + glucose	—	19.0 ± 0.0^b^	18.0 ± 0.0^c^	>90^c^	—	5.0 ± 0.0^ac^
	Galactose	—	18.0 ± 0.0^c^	20.0 ± 0.0^d^	19.0 ± 0.0^d^	—	4.0 ± 0.0^ac^

*L. casei *1020	Control	—	15.0 ± 0.0^a^	—	16.0 ± 0.0^a^	—	—
	Xylitol	10.0 ± 0.0^a^	16.0 ± 0.0^b^	ND	12.0 ± 1.4^b^	8.0 ± 0.0	8.5 ± 0.7^a^
	Galactosyl-xylitol	1.0 ± 0.0^b^	>90^c^	>90^a^	>90^c^	—	7.0 ± 0.0^a^
	Galactose + glucose	—	14.0 ± 0.0^d^	>90^a^	>90^c^	—	—
	Galactose	—	12.0 ± 0.0^e^	10.0 ± 0.0^b^	16.0 ± 0.0^a^	—	—

*L. paracasei* 0921	Control	—	11.0 ± 1.4^a^	—	10.5 ± 0.7^a^	—	—
	Xylitol	—	20.0 ± 0.0^b^	>90^a^	2.0 ± 0.0^b^	—	—
	Galactosyl-xylitol	—	>90^c^	>90^a^	7.0 ± 0.0^c^	—	—
	Galactose + glucose	—	5.0 ± 0.0^d^	2.0 ± 0.0^b^	8.0 ± 0.0^d^	—	—
	Galactose	—	3.0 ± 0.0^e^	8.0 ± 0.0^c^	2.0 ± 0.0^b^	—	—

*L. pentosus *0979	Control	—	32.5 ± 3.5^a^	—	8.0 ± 2.8^a^	4.0 ± 0.0	9.0 ± 1.4^a^
	Xylitol	15.0 ± 0.0^a^	>90^b^	15.0 ± 0.0^a^	10.0 ± 0.0^a^	—	—
	Galactosyl-xylitol	2.0 ± 0.0^b^	>90^b^	>90^b^	>90^b^	—	9.0 ± 0.0^a^
	Galactose + glucose	—	21.0 ± 0.0^c^	30.0 ± 0.7^c^	>90^b^	—	4.0 ± 0.0^b^
	Galactose	—	18.0 ± 0.0^d^	16.0 ± 0.0^d^	15.0 ± 0.0^c^	—	3.0 ± 0.0^c^

*L. plantarum *0982	Control	6.5 ± 2.1^a^	28.0 ± 0.0^a^	ND	5.0 ± 0.0^a^	—	3.0 ± 0.0^a^
	Xylitol	5.0 ± 1.4^a^	17.5 ± 0.7^b^	>90^a^	9.0 ± 0.0^b^	—	1.0 ± 0.0^b^
	Galactosyl-xylitol	>90^b^	>90^c^	>90^a^	>90^c^	—	4.0 ± 0.0^c^
	Galactose + glucose	—	18.0 ± 0.0^b^	>90^a^	28.0 ± 0.0^d^	—	—
	Galactose	—	9.0 ± 0.0^d^	>90^a^	7.0 ± 0.0^e^	—	—

SD^1^: standard deviation.

>90: total inhibition of indicator strain.

^a,b,c,d,e^Statistically significant difference, *p* < 0.05.

**Table 2:** Linear growth index and inhibition/stimulation rate according to Abbot's formula of cell-free supernatant after lactic acid fermentation of *Lactobacillus pentosus *0979 and *Lactobacillus paracasei *0921 towards *Alternaria brassicicola*.

LAB	Polyol/gal-polyol	Estimated value^*∗*^	Content of cell-free supernatant of LAB (v/v)					
			0%	10%	20%	30%	50%	70%
*L. pentosus* 0979	Xylitol	*T*	14.3	0	0	0	0	0
		*I* [%]	—	100	100	100	100	100
	Galactosyl-xylitol	*T*	26.6	0	0	0	0	0
		*I* [%]	—	100	100	100	100	100

*L. paracasei* 0921	Xylitol	*T*	6.4	5.6	1.8	0	0	0
		*I* [%]	—	12.5	71.9	100	100	100
	Galactosyl-xylitol	*T*	6.8	0	0	0	0	0
		*I* [%]	—	100	100	100	100	100

^*∗*^ *T*: linear growth index [—]; *I*: inhibition/stimulation rate according to Abbot's formula [%].
